The article "Analysis of the Effect of Laparoscopic and Open Surgical Treatment in Children with Congenital Megacolon" was retracted in 2023. Reasons: signs of a paper mill; suspected computer-generated content; unreliable results or conclusions; concerns about the data.

# Analysis of the Effect of Laparoscopic and Open Surgical Treatment in Children with Congenital Megacolon

**DOI:** 10.1155/2022/2669294

**Published:** 2022-06-08

**Authors:** Ziyi Chen, Bin Zheng, Hai Yang, Zhiwei Fang, Qiue Liu, Qingxiang Zheng

**Affiliations:** Department of Pediatric Surgery, Meizhou People's Hospital (Huang Tang Hospital), Meizhou, Guangdong Province 514000, China

## Abstract

In this paper, we have compared and analyzed the effect of laparoscopic and open surgical treatments in children with congenital megacolon. To address this, a total of 64 children with congenital megacolon who underwent surgery in the hospital, particularly from April 2014 to December 2020, were selected as the research objects. They were divided into control and observation groups by the random number table method, with 32 cases in each group. The control and observation groups were treated with open surgical and laparoscopic treatments, respectively. The treatment effects of the two groups were compared. The enema time, operation time, blood loss, anal defecation time, and duration of postoperative hospital stay of the observation group were lower than those of the control group. The comparison between the two groups was statistically significant (*P* < 0.05). There was no significant difference in CRP and WBC between the two groups before surgery (*P* > 0.05). The CRP level and WBC of the two groups were both increased after operation, the CRP level of the observation group was lower than that of the control group, the difference was statistically significant (*P* < 0.05), the WBC of the two groups was not statistically significant (*P* > 0.05). The rate of excellent and good defecation in the observation group on the 7th day after surgery was higher than that in the control group, and the difference was statistically significant (*P* < 0.05). There was no significant difference in Krickenbeck scores between the two groups before surgery (*P* > 0.05); 6 months after the surgery, the score of Krickenbeck in both groups increased, and that of the observation group was higher than that of the control group, indicating a difference in the overall score (*P* < 0.05). The total complication rate within 7 days after surgery in the observation group was lower than that in the control group, and the difference was not statistically significant (*P* > 0.05). Laparoscopic treatment of congenital megacolon could improve surgical indicators and reduce stress response in children, improve defecation and anal function, reduce the risk of complications, and promote recovery.

## 1. Introduction 

Congenital megacolon is a common clinical malformation of the digestive tract in children, also known as intestinal agangliocytosis [1]. The lack of ganglion cells in the colon of children leads to continuous intestinal spasm, which causes fecal deposition in the proximal colon and causes hypertrophy and expansion of the proximal colon, in turn, it causes constipation, malnutrition, colitis, and other problems, and the incidence is about 1/5000∼1/2000 [2, 3]. Congenital megacolon ranks in the forefront of neonatal intestinal malformation for many years and is clearly associated with the genetic inheritance of children. In the early clinical stage, it only manifests as loss of appetite, constipation, and abdominal distension [4]. The pathology is due to the lack of intermuscular ganglion in the diseased intestine, which leads to continuous spasm in the rectum or distal colon [5]. Radical surgery for congenital megacolon has gradually become matured after decades of development at home and abroad; among them, the relatively commonly used surgical methods include Swenson, Soave, and Duhamel. The traditional surgical methods have great trauma and bleeding, and the probability of complications is high [6, 7].

In this paper, we have compared and analyzed the effect of laparoscopic and open surgical treatments in children with congenital megacolon by selecting two different groups of children, i.e., control and observation. The control and observation groups were treated with open surgical and laparoscopic treatments, respectively. The results of laparoscopic treatment and open surgical treatment were observed and reported to verify our claim.

The rest of the paper is organized as follows.

In Section 2, basic materials of the proposed study, i.e., children and their selection and rejection criteria along with treatment plans are discussed in detail. Additionally, surgical details are also provided for both groups. In Section 3, various observation were presented and elaborated the effectiveness of the proposed study. Finally, concluding remarks are given.

## 2. Materials and Methods

### 2.1. Basic Materials

A total of 64 children with congenital megacolon who underwent surgery in our hospital from April 2014 to December 2020 were selected as the research objects. They were divided into the control group and observation group by the random number table method, 32 cases in each group. In the observation group, there were 18 boys and 14 girls. The age ranged from 3 months to 12 years, with an average of (38.9 ± 2.21) months. The body weight was 5.0∼34 kg, with an average of (13.1 ± 1.27) kg. There were 27 cases of normal type and 5 cases of short segment type. In the control group, there were 20 boys and 12 girls. The age ranged from 3 months to 12 years, with an average of (30.3 ± 1.13) months. The body weight was 5.7∼40 kg, with an average of (12.43 ± 2.36) kg. There were 22 cases of normal type and 2 cases of short segment type and 6 cases of long segment type. This study was approved by the hospital ethics committee. There was no significant difference in age, gender, disease type, and other general data between the two groups (*P* > 0.05).

### 2.2. Inclusion and Exclusion Criteria

#### 2.2.1. Inclusion Criteria

(1) “Expert consensus on diagnosis and treatment of congenital megacolon” diagnostic criteria [8]. (2) Age > 3 months. (3) There were symptoms of abdominal distension and constipation that were prolonged and difficult to recover. (4) The guardian of the children knew about this experiment and signed the informed consent.

#### 2.2.2. Exclusion Criteria

(1) Margin disease of megacolon. (2) Complicated with other congenital diseases. (3) Combined with other organ dysfunction. (4) Cannot tolerate this operation. (5) Cannot cooperate with the experiment.

### 2.3. Methodology

#### 2.3.1. Surgical Methods

Before surgery, three routine examinations, liver and kidney function, electrolyte, coagulation function, and hepatitis B were completed in the two groups. ECG examination can provide strong evidence for anemia and electrolyte disorder in seriously ill children. Antibiotics and warm saline enema were given 3 days before surgery, the fasting was started 1 day before the operation, there was metronidazole enema treatment on the day of operation, cephalosporin antibiotics were used 30 min before surgery, and routine preoperative fasting and catheterization were performed.

#### 2.3.2. Control Group

The children were under epidural anesthesia or general anesthesia, lying on their backs with high buttock, and lower extremities with sterile wrap after disinfection. The left lower abdominis rectus incision was made to expose the hypertropic intestinal segment, open the pelvic peritoneum, protect the ureter, ligate the blood vessels, free the intestinal canal, dilate the anus, clean the rectum, and keep the anus open. The excess anterior wall of the colon was removed, and the anterior wall of the anal canal was aligned with the posterior wall of the colon. The two forceps were clamped in an inverted V-shaped clamp with the ends of the two forceps crossed, and the two forceps were properly fixed [9]. A few days later, the intestinal wall of the clamps was necrotic and detached, and the proximal intestinal walls were conglutinated and healed, forming a new ampullary of the rectum.

#### 2.3.3. Observation Group

An incision was made through the umbilical hole, trocars (5 mm) were placed to create a pneumoperitoneum, and trocars (5 mm) were placed in the right lower abdomen and left middle abdomen, respectively, as the operation holes. The colon was lifted, the mesentery was exposed, and the mesangial vascularized area was opened with an ultrasound knife to cut off the tertiary vascular arch; pulled out of the colon to the anal orifice without tension, cleared no bleeding, and relieved pneumoperitoneum. The rectal mucosa was cut 0.5∼1.0 cm in the dentate line, the traction line was sutured, and the rectal mucosa was dissected. The full layer and anterior mucosa of the posterior wall of the rectum were removed. The pneumoperitoneum was reconstructed, the abdominal cavity was explored, and the colon was confirmed to have no tension, torsion, internal hernia, bleeding, and organ damage when pulled down [10]. Both groups received conventional anti-infection treatment after operation.

### 2.4. Evaluation Criteria

#### 2.4.1. Operation Indicators

The enema time, operation time, blood loss, anal defecation time, and duration of postoperative hospital stay were compared between the two groups.

#### 2.4.2. Stress Response Indicators

Fasting venous blood of 5 ml was collected before and 1 d after surgery, respectively. The white blood cell count (WBC) of 2 groups was measured by using the Sysmex F-800 automatic blood cell analyzer in one group. The other one was centrifuged at 3000 r min^−1^ for 10 min, the supernatant was taken, and the serum C-reactive protein (CRP) level of the two groups was determined by the enzyme-linked immunosorbent assay [11].

#### 2.4.3. Condition Defecation

According to the Zakaria scale [12], the defecation of the child was determined. (1) Score for defecation frequency: 2 points was for defecation frequency ≥1 times a day, 1 point was for defecation frequency ≥3 times a week, and 0 point was for defecation frequency <3 times a week. (2) Bloating score: 2 points was for no bloating, 1 point was for occasional bloating, and 0 point was for frequent bloating. ③ Fecal fouling score: 4 was for unfouled feces, 3 was for less than 3 times per week, 2 was for more than 3 times per week, 1 was for loose stool incontinence, and 0 was for complete stool incontinence. Project score: 7∼8 was excellent; 5∼6 was good; 3∼4 was general; 0 to 2 was bad. Excellent and good rate = (excellent case number + good case number)/total case number of the group × 100%.

#### 2.4.4. Anus Function

Krickenbeck score was used to evaluate children's anal function, including constipation, fecal fouling, and intestinal voluntary peristalsis, with a total score of 0∼9. The higher the score, the better the anal function.

#### 2.4.5. Complication Rate

The complications of the two groups were compared.

### 2.5. Observation Index

The differences in operation time, blood loss, anal defecation time, and duration of postoperative hospital stay between the two groups were compared. The incidence of complications within 7 days after surgery and the difference of defecation on 7 days after surgery were observed.

### 2.6. Statistical Method

The SPSS 20.0 statistical software was used for data analysis. Measurement data were expressed as mean ± standard deviation (*x* ± *s*) and compared by *t*-test; The enumeration data were presented as percentage (%), and the *χ*^2^ test was used for comparison. *P* < 0.05 was considered statistically significant.

## 3. Results and Observations

### 3.1. Operation Indicators

The enema time, operation time, blood loss, anal defecation time, and duration of postoperative hospital stay of the observation group were lower than those of the control group, and the comparison between the two groups was statistically significant (*P* < 0.05). Comparison of operation indicators of two groups was shown in Table 1.

### 3.2. Stress Response Indicators

There was no significant difference in CRP and WBC between the two groups before surgery (*P* > 0.05); The CRP level and WBC of the two groups were both increased after operation, the CRP level of the observation group was lower than that of the control group, the difference was statistically significant (*P* < 0.05), and the WBC of the two groups was not statistically significant (*P* > 0.05). Comparison of stress response indicators of two groups is shown in Table 2.

### 3.3. Condition Defecation

The rate of excellent and good defecation in the observation group on the 7th day after surgery was higher than that in the control group, and the difference was statistically significant (*P* < 0.05). Comparison of condition defecation of two groups is shown in Table 3.

### 3.4. Anus Function

There was no significant difference in Krickenbeck scores between the two groups before surgery (*P* > 0.05); 6 months after the surgery, the score of Krickenbeck in both groups increased, and that of the observation group was higher than that of the control group, indicating a difference in the overall score (*P* < 0.05). The comparison of the anus function of the two groups is shown in Table 4.

### 3.5. Complication Rate

The total complication rate within 7 days after surgery in the observation group was lower than that in the control group, and the difference was not statistically significant (*P* > 0.05). Comparison of complication rate of two groups is shown in Table 5.

## 4. Discussion

There are many surgical treatments for congenital megacolon, for example, each operation is different in the way of excision of intestinal canal, the treatment of nonganglion intestinal segment or postoperative additional operation [13]. In pediatric children, the most common disease is the congenital megacolon. More specifically, it is defined as a condition for which cause is unknown and is usually described by ganglion cells. The main clinical manifestation is intestinal obstruction, which can cause malnutrition and even enteritis, seriously endangers the growth and development of children [14]. Therefore, the clinical treatment should be selected in time to control the disease and ensure the healthy growth and development of children [15]. The lack of ganglion cells in the colon of children leads to continuous intestinal spasm, which causes fecal deposition and proximal colon hypertrophy and expansion, which in turn leads to constipation, vomiting, abdominal distension, developmental delay, and other problems [16]. Although transanal megacolon radical surgery can effectively remove the lesions and relieve the clinical symptoms, the risk of postoperative colon stenosis, constipation, infection, and other occurrence is high, so the application has certain limitations [17]. Laparoscopic-assisted radical transanal megacolon surgery is a minimally invasive operation where posterior peritoneum is not separated to obtain a clear field of vision. The incision is small; hence, it can reduce the amount of bleeding, reduce trauma, and speed up postoperative recovery [18]. In addition, with the aid of laparoscopy, it can realize effective detection, prevent excessive pulling, and prevent fecal infection [19].

This study showed that the enema time, operation time, blood loss, anal defecation time, and duration of postoperative hospital stay of the observation group were lower than those of the control group, and the comparison between the two groups was statistically significant (*P* < 0.05). There was no significant difference in CRP and WBC between the two groups before surgery (*P* > 0.05). The CRP level and WBC of the two groups were both increased after operation, the CRP level of the observation group was lower than that of the control group, the difference was statistically significant (*P* < 0.05), and the WBC of the two groups was not statistically significant (*P* > 0.05). The rate of excellent and good defecation in the observation group on the 7th day after surgery was higher than that in the control group, and the difference was statistically significant (*P* < 0.05). There was no significant difference in Krickenbeck scores between the two groups before surgery (*P* > 0.05); 6 months after the surgery, the score of Krickenbeck in both groups increased, and that of the observation group was higher than that of the control group, indicating a difference in the overall score (*P* < 0.05). The total complication rate within 7 days after surgery in the observation group was lower than that in the control group, and the difference was not statistically significant (*P* > 0.05).

## 5. Conclusion

In this paper, we have compared and analyzed the effect of laparoscopic and open surgical treatments in children with congenital megacolon by selecting two different groups of children, i.e., control and observation. Laparoscopic treatment of congenital megacolon has the capacity to improve surgical indicators and reduce stress response in children, improve defecation and anal function, reduce the risk of complications, and promote recovery.

## Figures and Tables

**Table 1:** Comparison of operation indicators of two groups.

Operation indicators	Observation group	Control group	*t*	*P* value
Enema time (d)	15.8 ± 1.15	14.68 ± 1.53	−0.926	<0.05
Operation time (min)	148.60 ± 33.42	148.40 ± 36.41	−4.344	<0.05
Blood loss (mL)	6.37 ± 1.45	18.84 ± 2.36	−7.815	<0.05
Anal defecation time (d)	2.56 ± 1.01	2.84 ± 1.14	0.578	<0.05
Duration of postoperative hospital stay (d)	8.93 ± 2.18	10.37 ± 2.57	−1.112	<0.05

**Table 2:** Comparison of stress response indicators of two groups.

Groups	CRP/(mg • L^−1^)		WBC/(×10^9^L^−1^)	
	Before surgery	1 day after surgery	Before surgery	1 day after surgery
Observation group	1.22 ± 0.41	17.45 ± 9.52	7.87 ± 1.84	12.07 ± 3.31
Control group	1.02 ± 0.51	31.02 ± 7.35	8.74 ± 2.03	12.70 ± 4.27
*T*	0.904	2.753	0.438	0.786
*P* value	>0.05	<0.05	>0.05	>0.05

**Table 3:** Comparison of condition defecation of two groups.

Groups	Excellent	Good	General	Bad	Excellent and good defecation
Observation group	27 (84.38)	3 (9.38)	1 (3.12)	1 (3.12)	30 (93.75)
Control group	18 (56.25)	7 (21.88)	3 (9.38)	4 (12.50)	25 (78.12)
*P* value					<0.05

**Table 4:** Comparison of anus function of two groups.

Groups	Before surgery	6 months after surgery	*t*	*P* value
Observation group	3.25 ± 0.41	7.84 ± 0.71	33.731	<0.05
Control group	3.34 ± 0.52	7.06 ± 0.54	30.072	<0.05
*T*	0.886	5.217		
*P* value	>0.05	<0.05		

**Table 5:** Comparison of complication rate of two groups.

Groups	Bleeding	Infection	Intestinal obstruction	Total complication rate
Observation group	1 (3.125)	1 (3.125)	1 (3.125)	3 (9.375)
Control group	1 (3.125)	6 (18.75)	2 (6.25)	9 (28.125)
*χ* ^2^	0.452	0.521	0.511	0.204
*P* value	>0.05	>0.05	>0.05	>0.05

## Data Availability

The data used to support the findings of this study are included within the article.
